This article has been retracted.

# Is insulin resistance the cause of fibromyalgia? A preliminary report

**DOI:** 10.1371/journal.pone.0216079

**Published:** 2019-05-06

**Authors:** Miguel A. Pappolla, Laxmaiah Manchikanti, Clark R. Andersen, Nigel H. Greig, Fawad Ahmed, Xiang Fang, Michael A. Seffinger, Andrea M. Trescot

**Affiliations:** 1 Department of Neurology, University of Texas Medical Branch, Galveston, Texas, United States of America; 2 St. Michael’s Pain & Spine Clinics, Houston, Texas, United States of America; 3 Department of Anesthesiology, LSU School of Medicine Health Sciences Center, New Orleans, Louisiana, United States of America; 4 Office of Biostatistics, University of Texas Medical Branch, Galveston, Texas, United States of America; 5 Drug Design and Development Section, National Institute on Aging, National Institutes of Health, Bethesda, Maryland, United States of America; 6 Department of Neuromusculoskeletal Medicine, College of Osteopathic Medicine of the Pacific, Pomona, California, United States of America; 7 Pain and Headache Center, Eagle River, Alaska, United States of America; Henan University of chinese medicine, CHINA

## Abstract

Fibromyalgia (FM) is one of the most frequent generalized pain disorders with poorly understood neurobiological mechanisms. This condition accounts for an enormous proportion of healthcare costs. Despite extensive research, the etiology of FM is unknown and thus, there is no disease modifying therapy available for this condition. We show that most (if not all) patients with FM belong to a distinct population that can be segregated from a control group by their glycated hemoglobin A1c (HbA1c) levels, a surrogate marker of insulin resistance (IR). This was demonstrated by analyzing the data after introducing an age stratification correction into a linear regression model. This strategy showed highly significant differences between FM patients and control subjects (p < 0.0001 and p = 0.0002, for two separate control populations, respectively). A subgroup of patients meeting criteria for pre-diabetes or diabetes (patients with HbA1c values of 5.7% or greater) who had undergone treatment with metformin showed dramatic improvements of their widespread myofascial pain, as shown by their scores using a pre and post-treatment numerical pain rating scale (NPRS) for evaluation. Although preliminary, these findings suggest a pathogenetic relationship between FM and IR, which may lead to a radical paradigm shift in the management of this disorder.

## Introduction

Fibromyalgia (FM) is one of the most frequent generalized pain disorders with poorly understood neurobiological mechanisms. In the general population, the estimated global prevalence of FM is 2.7% with a 3 to 1 female to male ratio [1]. However, studies suggest an even higher prevalence in primary care settings [2].

Patients afflicted with FM have chronic widespread pain and protean somatic symptoms including fatigue, nonrestorative sleep, gastrointestinal complaints and problems of cognition and mood [3].

The global economic impact of FM is enormous. In the United States alone, the healthcare cost is around $100 billion/year; comparable to reports in European countries [4]. Due to lower pain thresholds, patients with FM also have a higher incidence of symptomatic musculoskeletal and spinal disorders, which in themselves contribute to the financial burden of managing this disorder.

FM is considered a central sensitivity pain disorder characterized by abnormal processing of nociceptive stimuli [5]. In addition, peripheral mechanisms (see Discussion below regarding small fiber neuropathy) are also believed to contribute to widespread pain.

Many hypotheses have been advanced to explain the extensive array of symptoms including inherited abnormalities [6], dysfunction of neurotransmitter pathways such as substance P [6], immune dysregulation [7–9] and several others [9]. Unfortunately, none of these propositions has led to practical advances beyond symptomatic treatment. In fact, recent reviews of FM published in 2016 [10] and 2017 [3], have concluded that there have been no substantive advances in our understanding of this disease.

Prior observations indicate that IR causes dysfunctions in the brain microvasculature leading to focal cerebral hypoperfusion [11]. Since similar brain perfusion abnormalities are present in patients with FM [12], we hypothesized that IR may be the missing link in this disorder. In order to search for initial evidence in support of this hypothesis, we conducted a retrospective chart review of patients with FM focusing on potential laboratory abnormalities. In contrast with prior studies, when we applied an age correction to the data available for analysis, specifically to the HbA1c values, unexpected findings came to light. Here, we report that a series of patients with FM belong to a distinct population that can be segregated from a control group by their HbA1c values, a biomarker for impaired glucose metabolism, characterized by insulin resistance [13, 14].

In order to supplement this finding, we also reviewed the evolution of the pain scores of patients with FM who had had their IR treated pharmacologically. This subgroup of patients reported dramatic improvements of their myofascial pain after treatment with metformin.

This evidence, although preliminary, suggests a pathogenetic relationship between FM and IR, which may lead to a paradigm shift in the management of this disorder.

## Materials and methods

### Sample description

We identified 23 patients from a retrospective chart review who were referrals to a subspecialty pain medicine clinic for the treatment of widespread myofascial pain. All patients had met the 1990 [15] as well as the 2010/2011 [16] American College of Rheumatology criteria for FM diagnosis (i.e., tender points were retained in the evaluation). Patients with comorbid disorders, including history of cerebrovascular disease, rheumatoid arthritis, untreated endocrine abnormalities, autoimmune conditions, neuromuscular diseases, active malignancy, immunodeficiency or drug or alcohol abuse were excluded from the sample. Patients taking medications associated with IR such as glucocorticoids, thiazide diuretics, atypical anti-psychotics, beta-blockers, niacin, statins and others were also excluded.

Since there is a known association between small fiber neuropathy and FM [17, 18], many of these patients had undergone laboratory investigations in commercial CLIA (United States Clinical Laboratory Improvement Act) accredited laboratories. This comprised diagnostic panels for peripheral neuropathy, which included HbA1c values.

The HbA1c values from 23 patients with FM (8 Hispanic; 11 White; 4 African-American; 21 females, 2 males) were compared with the HbA1c means of two independent control populations. One was a non-diabetic population with normal glucose tolerance (obtained from the Framingham Offspring Study; FOS NGT) for the ages stated in the graph (Fig 1). The second population used for confirmation was extracted from the National Health and Nutrition Examination Survey dataset (NHANES non-diabetic) available from the Centers for Disease Control and Prevention (CDC). The data from both control groups can be found published in Pani et al [19].

**Fig 1:** HbA1c in patients with fibromyalgia versus controls.

Because peripheral neuropathies (including small fiber neuropathy) that are associated with IR may start at very early stages of pre-diabetes, there is a growing trend among experts to begin early pharmacological interventions to correct this abnormality, particularly when IR is associated with neuropathy or other risk factors [20]. Following this premise, patients either meeting criteria for pre-diabetes (HgA1c values of 5.7 or higher) or previously undiagnosed diabetes mellitus type 2, are routinely offered treatment in our clinics and were initiated on metformin 500 mg twice a day. In our sample of patients, metformin was added to “standard treatment” for widespread myofascial pain. Standard treatment (ST) consisted of either norepinephrine reuptake inhibitors (amitriptyline, duloxetine or milnacipran) and/or membrane stabilizing agents (gabapentin or pregabalin), depending on tolerability or patients’ preference of either class of drug. In our clinics, pain scores are routinely recorded by the Numeric Pain Rating Scale (NPRS), at each clinical encounter. The NPRS is a unidimensional measure of pain intensity in adults which consists of an 11-point scale for self-reporting of pain. It is one of the most commonly employed instruments in clinical and research settings with extensive evidence supporting its validity [21]. Pain scores were available from the initial evaluation, after ST and after metformin administration.

### Statistical analyses

In order to characterize the variation contributed from the patients, sets of simulated HbA1c data were generated to emulate the populations which were the source of the HbA1c values in the controls. Separately for FOS NGT and NHANES nondiabetic, over the bounded age range from 40 to 69, the tabled values of N, mean, and standard error of each age group were used to estimate the corresponding standard deviation (estimating standard deviation for each age group as the product of the standard error and square root of N). A corresponding simulated source population for the data was generated for each centered age as a set of random normally distributed values with the tabled Ns and means and the calculated standard deviation (Table 1). Means and standard errors for the resulting simulated data over each age range were verified in good agreement with the values, with estimates of means within 0.1% and standard errors within 4%. This simulated FOS NGT and NHANES non-diabetic HbA1c data, paired with the HbA1c measures from patients with FM, was then modeled by linear regression with relation to age and group (FOS HGT simulated patients (N = 1350), NHANES nondiabetic simulated patients (n = 1592) versus FM patients (n = 23). Differences among the groups were estimated by Tukey-adjusted contrasts (Table 2). Differences among pain scores (initial, ST-NPRS, MET-NPRS) were pairwise estimated using the sign test, followed by Hommel adjustment of p-values to compensate for multiple comparisons. Statistical analyses were performed using R statistical software (R Core Team, 2018, version 3.5.1). All statistical tests assumed a 95% level of confidence, with alpha = 0.05.

**Table 1:** 

	Estimate	SE	p-value
NHANES Nondiabetic—FOS NGT	0.20	0.02	< 0.0001
Fibromyalgia—FOS NGT	0.59	0.1	< 0.0001
Fibromyalgia—NHANES Nondiabetic	0.39	0.1	0.0002

Differences in HbA1c among groups, per Tukey-adjusted differences from regression model.

**Table 2:** 

	Median	Min	Q1	Q3	Max
Initial	8	5	6.75	8	8
ST- NPRS	4	2	3	4.25	8
MET—NPRS	0.25	0	0	0.5	2

Numerical Pain Rating Scores. All pairwise differences among the groups were significant, p < 0.0001, per the sign test and following adjustment for multiple comparisons.

This study has been determined by an Investigational Review Board (Integreview, Austin, TX) to meet the exempt criteria according to the Code of Federal Regulations governing the performance of this research.

## Results

### 1. Association between FM and HbA1c levels

From all analytes reviewed, only the HbA1c levels segregated patients with FM from control subjects (Fig 1). Despite many patients with FM showing HbA1c values within the normal range (equal or less than 5.6%), when we stratified the data in an age continuum and analyzed it as described, a clear-cut difference between the groups (patients with FM versus controls) came to light. The regression relating HbA1c to group (FOS NGT, NHANES nondiabetic, fibromyalgia HbA1c), summarized in Fig 1 and Table 1, showed that patients with FM average 0.59 units of HbA1c higher than FOS NGT, p < 0.0001, and that patients with FM average 0.39 units higher than NHANES nondiabetic, p = 0.0002.

NPRS for patients who were treated with metformin are reported in graphic form in Fig 2.

**Fig 2:** Effect of metformin treatment on pain as measured by the NPRS (0–10 scale).

Pain scores differed significantly per the sign test among all groups (initial, ST-NPRS, MET-NPRS), with p <0.0001 in each pairwise comparison, as illustrated in Fig 2 and summarized in Table 2.

HbA1c values in 23 patients with FM (8 Hispanic; 11 White; 4 African-American; gender: 21 females, 2 males) were compared with the means of two control populations as described in the text. 1-A non-diabetic population with normal glucose tolerance (obtained from the Framingham Offspring Study) and 2-A nondiabetic population from the NHANES data set. Regression lines are shown with shaded 95% confidence regions. FOS NGT and NHANES nondiabetic HbA1c values include scatterplots of published mean values for each age region, while HbA1c results from patients with FM include a scatterplot of measures from individual patients (several overlap in values). The regression estimates that HbA1c values in patients with FM average 0.59 +/- 0.1 (mean +/-SE) units higher than FOS NGT (p<0.001), and 0.39 units higher than the NHANES nondiabetic values, p = 0.0002. Because of overlapping values, not all individual patients can be plotted in the graph. For this reason, individual data values for each patient are provided in Table 3.

**Table 3:** 

Age	HbA1c	I-NPRS	ST-NPRS	M-NPRS	LMT-M
35	5.1% (32 mmol/l)				
36	5.7% (39 mmol/l)	8	4	0	15
38	5.5% (37 mmol/l)				
43	5.4% (36 mmol/l)				
43	5.7% (39 mmol/l)	7	3	1	16
45	5.2% (33 mmol/l)				
45	5.8% (40 mmol/l)	8	5	2	25
46	5.7% (39 mmol/l)	8	4	2	12
46	5.7% (39 mmol/l)	8	3	1	12
47	5.5% (37 mmol/l)				
49	6.1% (43 mmol/l)	8	8	0	24
49	5.4% (36 mmol/l)				
51	5.9% (41 mmol/l)	8	4	0.5	10
52	5.7% (39 mmol/l)				
53	6.5% (48 mmol/l)	6	2	0	24
54	6.0% (42 mmol/l)	5	5	0	36
54	6.0% (42 mmol/l)	7	3	0	8
56	5.7% (39 mmol/l)	7	3	0.5	36
58	5.8% (40 mmol/l)	5	2	0	8
60	6.1% (43 mmol/l)	6	2	0.5	12
59	5.8% (40 mmol/l)	8	3	0.5	12
51	6.0% (42 mmol/l)	8	4	1	12
46	6.1% (43 mmol/l)	8	4	0	12

Depicted are individual patients’ age, HbA1c % with corresponding mmol/l between parenthesis, pain scores at initial encounter (I-NPRS), pain scores after standard treatment (ST-NPRS), pain scores after metformin treatment (M-NPRS) and length of metformin treatment in months (LMT-M). Patients retained the therapeutic effect of metformin at the time of their last clinical encounter as indicated in LMT-M.

### 2. Pain scores reduction after treatment of IR

The subgroup of patients who had undergone pharmacological treatment of IR with metformin, in combination with the ST, experienced a dramatic decrease in the pain scores (Fig 2). Response to metformin plus ST was followed by complete resolution of the pain (report of 0 of 10 in the NPRS) in 8 of 16 patients who had been treated with metformin (50%), a degree of improvement never observed before in such a large proportion of FM patients subjected to any available treatment. In contrast, patients treated with ST alone improved, but complete resolution of pain was generally not observed (Fig 2). Interestingly, some patients responded *only to metformin* and not to ST with NSRIs or membrane stabilizing agents. Importantly, there was a long-term retention of the analgesic effect of metformin as noted in Table 3.

I-NPRS: Initial pain scores at presentation. 2-ST-NPRS: Numerical pain scores after standard treatment (pregabalin, gabapentin and/or NSRIs). M-NPRS: Numerical pain scores after addition of metformin. Pain scores are the average of the worse pain experienced in the 7 days prior to the encounter. All pairwise differences among the groups were significant, p<0.0001, per the sign test and following adjustment for multiple comparisons, as shown in Table 2.

## Discussion

The results showed a highly significant association between FM and HbA1c levels. Stratification of the values in an age continuum, showed a clear-cut difference between the patients and the control groups. As can be visually appreciated in the graph in Fig 1, almost all patients in the FM group fell at or above the mean of the FOS control values, with highly significant differences between the FM patients and both control groups (p < 0.0001 and p = 0.0002 for the FOS and NHANES control populations, respectively). In addition, patients with FM in whom IR had been pharmacologically treated showed dramatic and statistically significant reductions in pain scores (p < 0.0001 for all groups) as shown in Fig 2 and Tables 2 and 3.

HbA1c does not directly measure IR; however, it is widely recognized as a surrogate marker for this abnormality [14]. Non-diabetic individuals with mildly elevated HbA1c values (5.7%-6.4%), belong to a stage often called “pre-diabetes”, which carries a higher risk for the development of peripheral neuropathies (15), cardiovascular events [13], neurological disease [22–24] and all-cause mortality [13].

In view of the substantive research efforts involved in FM, including those from the pharmaceutical industry, we were puzzled that prior investigations had overlooked these simple findings. The main reason for this oversight is that many patients with FM show HbA1c values currently considered to be within the normal range; however, this is the first study to analyze the data in an age-stratified manner. This is important, considering the effect of aging on HbA1c levels [19]. Therefore, a value of 5.5%, for example (considered “normal” by current criteria), may not be so in many young subjects. An additional reason for having missed this association may be as follows: prior studies have established an association between FM and small fiber neuropathy [17, 18]. Although IR is a frequent cause of small fiber neuropathy, work up of this disorder by the investigators of these studies did not include evaluation of HbA1c levels. Instead, other methods were used in some studies [i.e., oral glucose tolerance tests; for example, see [17]]. Our data, if confirmed, may explain not only mechanisms germane to central pain in FM but also, the association between this disorder and small fiber neuropathy.

It is important to give credit to the effort of other investigators who have also sought this association. Tishler et al [25] found that the incidence of FM was higher in patients with diabetes mellitus type 2 than in their control group (18% versus 2%) and suggested a potential relationship between these two disorders. In a separate study, Yanmaz et al [26] reported similar findings.

Fava et al [27] showed that IR was a risk factor for cognitive impairment in FM patients, but this association was limited only to cognitively impaired patients. These results would be problematic for any causative hypothesis because, one cannot claim causation for a factor that is present only in a small subgroup of the population afflicted by the condition. However, by applying the strategy for data analysis reported in this study, we now demonstrate that abnormalities likely related to IR are much more widespread than had previously been appreciated and may be present in most (and perhaps all) patients with FM. Interestingly, in the study from Fava et al [27], the subjects body mass index and waist-to-hip ratio were not associated with an increase in their risk for developing cognitive impairment, suggesting that the occurrence of IR in these patients may not necessarily be associated with the increased body mass index often present in patients with FM [28].

Based on our data, we would like to propose that IR is pathogenetically linked to FM. However, there are several caveats to our proposition which must be carefully considered in the design of future clinical trials attempting to confirm this hypothesis. One is the limitation intrinsic to retrospective cross-sectional studies. Because IR and FM were simultaneously assessed, evidence for causality is more difficult to establish in the absence of a temporal relationship. Secondly, patients with FM are commonly overweight or obese [28], factors which may predispose them to the development of IR [29]. Thirdly, the results of the pharmacological intervention were extracted from retrospective observations of treated patients and interpreted outside the context of a randomized placebo controlled clinical trial. Finally, metformin may have an effect in chronic pain *independent* of its action on IR [30, 31]. Metformin is known to increase mitochondrial AMPK [32–34] which can result in reduced mechanical allodynia and nociceptor activation [32–34]. In fact, one other group suggested that metformin may be useful in FM, although a relationship to IR was not suspected or investigated by the authors [35, 36]. In this regard, it would be important for future trials to include drugs that target IR by different mechanisms from metformin. Finally, other markers of IR, such as the homeostasis model assessment for insulin resistance (HOMA-IR) [37] and related tests should also be explored using similar analytic strategies for age correction and comparison with normal individuals. In their study, Fava et al [27] could not find differences between this test (HOMA-IR) in patients with FM when compared to a control population; however, no age corrections (as reported here) were applied to the comparison.

Despite all these caveats, this initial report prompts us to seek answers to a challenging set of questions generated by this hypothesis. It would be unlikely for a placebo type of effect alone to result in the impressive degree of long-lasting pain improvement experienced by the patients who received the drug combination (metformin plus ST). Remarkably, “non-responders” were conspicuously absent in our patient’s sample; such an unusual and atypically low “number needed to treat” (NNT) would be more in line with a disease modifying therapy.

In conclusion, IR is being increasingly associated with a broad number of neurological disorders [22–24] and FM may be one additional condition. Our data provides preliminary evidence suggesting that IR may be a pathological substratum in FM and sets the stage for future studies to confirm these initial observations. If confirmed, our findings may translate not only into a radical paradigm shift for the management of FM but may also save billions of dollars to healthcare systems around the world.
